# Evaluation of Cyclic Fatigue Resistance of Novel Replica-Like Instruments in Static Test Model

**DOI:** 10.1155/2024/8842478

**Published:** 2024-08-21

**Authors:** Uğur Aydın, Melih Özdemir, Emre Çulha, Muazzez Naz Baştürk Özer, Bilal Turan

**Affiliations:** Department of Endodontics Gaziantep University, Gaziantep, Türkiye

## Abstract

**Introduction:**

The aim of our study is to comparatively analyze the canal cyclic fatigue resistance of widely used rotary file systems, including EndoArt Touch Gold (ETG), Perfect MTF Plus Gold (PPG), Fanta V-Taper Gold (FVG), and ProTaper Next (PTN).

**Methods:**

Stainless steel canals with a 60° angle and a 3-mm curvature radius were specially prepared. The canals were shaped with each rotary file system and tested for resistance using a cyclic fatigue testing apparatus. The number of fracture cycles (NFC; K file tip separation) was measured. Data were analysed by one-way ANOVA and post hoc LSD tests.

**Results:**

PTN and PPG rotary file systems exhibited the highest NFC. The NFC value for PTN was 589 ± 63, and for PPG, it was 507 ± 51.

**Conclusion:**

The results of this study demonstrate that rotary file systems such as PTN and PPG exhibit higher cyclic fatigue resistance. ETG and FVG rotary file systems also possess generally acceptable cyclic fatigue resistance levels.

## 1. Introduction

Despite the advances in manufacturing of nickel–titanium (Ni–Ti) instruments, fracture of these instruments in root canals is still a matter of concern. Fatigue-related fracture commonly occurs either cyclic or torsional. Torsional fractures are related to stresses generated along the instrument simultaneous binding the tip of the instrument and continuing the remaining portion to rotate [1]. To reduce these stresses leading to torsional fractures, lubrication characteristics of irrigation agents may be beneficial [2]. On the other hand, cyclic fatigue fractures result from the tensile and compressive stresses subsequent to the repetitive use of instruments in narrow and curved canals [3]. Fractured instruments obstruct root canals and avoid adequate disinfection and thus may severely decrease the success rate if they are not removed from root canal system [4]. A number of factors influence the metallic fatigue of Ni–Ti rotary instruments. These include instrument design, metallurgical features, motion style of the instruments (rotation and reciprocation), operators' skill and experience, preparation technique, number of uses of the instrument, and number of sterilization cycles [5]. Additionally, anatomical condition of the canals, particularly in middle and apical regions of curved canals, may vary and influence fracture resistance of instruments which can be compensated by the operator's preoperative evaluation [6]. Thus, in vitro studies are more prone to achieve standardized evaluations.

Up to date several manufacturing methods have been developed including electro-polishing, production of heat treated wires so called M-wire, controlled memory- (CM-) wire, R-phase wire, different cross-sectional designs, and blue and gold plating to reduce the risk of instrument fractures [7, 8, 9]. Numerous previous studies comparatively evaluated the cyclic fatigue resistance of novel widely used Ni–Ti instruments and stated that different manufacturing methods increased the fatigue resistance of the instruments [8, 10, 11, 12].

ProTaper Next (PTN; Dentsply-Sirona, Ballegiues, Switzerland) is one of these popular instruments manufactured from M-Wire Ni–Ti alloy providing increased resistance and flexibility [9]. Its cross section geometry is rectangular in shape. This instrument rotates with its unique eccentric motion style providing only two corners touch canal walls during instrumentation and by this way decreasing friction. In previous studies, its resistance was compared with other novel popular instruments [7, 8, 13].

New trend in endodontics is the duplication of Ni–Ti rotary systems and their commercial availability to clinicians. These replica systems are often sold at lower prices than original rotary systems and have been widely used. However, their comparison with popular systems is limited in the literature remaining their resistance unclear. Three of these systems are EndoArt Touch Gold (ETG; Inci Dental, İstanbul, Turkey), Perfect MTF Plus Gold (PPG; Perfect Medical Instruments, Shenzhen, China), and Fanta V-Taper Gold (FVG; Fanta Dental, Shenzhen, China).

ETG is a Ni–Ti rotary system specifically designed for endodontic preparation, making canal preparation faster, effective, and safer. ETG files with convex triangular cross section are manufactured from CM-wire and further coated with gold plating which increases the cyclic fatigue resistance and flexibility.

PPG is a rotary system designed to provide faster, safer, and more consistent canal preparations with the ability to effectively shape root canals and optimize the canal preparation process. PPG system is made of Ni–Ti files produced with M-wire technology. Cutting edge efficiency is increased by using a rectangular cross section with eccentric motion. With its gold surface coating, it minimizes the friction of the file against the canal walls by reducing the friction and thus increases the cutting efficiency.

FVG is a six-file system including three S-files manufactured with AF™-R wire technology and three F-files manufactured with AF™-H wire technology. The manufacturer claims this production technology increases both flexibility and resistance. FVG files have a V-shaped design, so they better fit the natural anatomy of the canal. This allows the canal walls to be prepared more evenly, thus enabling more effective removal of all tissues and inflammatory debris within the canal. Additionally, this design minimizes potential damage during the canal preparation process and preserves the natural anatomy of the root canal. Gold plating helps FVG files reduce friction, allowing them to interact with the canal walls with less resistance. Additionally, less resistance prevents the file from overheating which extends the life of the file and reduces the risk of fracture. The extremely flexible wire structure of F1, F2, and F3 files gives them the “memory file” feature.

Although clinicians widely use replica rotary file systems, their mechanical performance has not been adequately evaluated sufficiently. To the best of our knowledge, there is no previous study evaluating cyclic fatigue of ETG, PPG, and FVG systems. The aim of this study is to evaluate the three low-priced replica Ni–Ti rotary file systems (ETG, PPG, and FVG) versus PTN in terms of cyclic fatigue. Our null hypothesis is that there will be no statistical difference regarding these parameters between four different rotary systems.

## 2. Materials and Methods

Sample size and power for statistical testing by a three-way analysis of variance were calculated a priori using *G* ^*∗*^Power (version 3.1.2, Heine Heinrich University, Dusseldorf, Germany). A sample size of 15 instruments in each group was determined to provide a power of 0.80 (*b* = 0.20) for detecting a mean difference that was 0.4 standard deviation in magnitude (*a* = 0.05). Before the test procedure, included instrument were inspected under a stereomicroscope with at ×20 magnification to exclude any file with a possible manufacturing defect. Fifteen size 25/06 instruments from each of the four tested systems were included. The test was performed with a static test model which uses a custom-made stainless steel block containing a curved artificial canal with an inner diameter of 1.5 mm, a curvature angle of 60°, and a radius of curvature of 3 mm (Figure 1). During testing, the handpiece was fixed using a holding arm. This fixed system enabled the files to operate with an endodontic motor (VDW Silver, VDW GmbH, Munich, Germany) at a speed of 300 rpm and a torque of 2 N/cm for all systems as recommended (Figure 2). The working length of each file was determined as 18 mm. The front of the stainless steel block was covered with glass to observe the moment when the files broke and to protect them from coming out of the artificial canals. Sodium hypochlorite was injected through the artificial canal orifices in each test group to control friction inside the canal. All files were operated within the artificial canal until file fracture occurred. The time until fracture occurred for each file was recorded in seconds with a stopwatch. The number of cycles to fractures (NCF) was calculated by multiplying the rotation speed (300 rpm for each according to the manufacturers) and the time (min).

The following formula was used to convert these breaking times into number of laps:

(1) $$\begin{array}{c} \text{NCF }=\;\frac{\text{Time to breakage }\left(s\right)\times \text{rotation speed of the file }\left(\text{rpm}\right)}{60}. \end{array}$$

Because the tested files were kept in a stable position at 18 mm length, the length of fractured segments was not measured.

Randomly selected fractured surfaces from each group was examined under scanning electron microscope with both ×200 and ×1,000 magnifications (SEM; JSM-6390, Jeol ABD Inc., Massachusetts, USA; Figure 3). As the inspection of the cross section geometry of ETG group was not in compliance with manufacturer's information, three more samples belong to this group were examined in order to verify the results (Figure 4).

Statistical analyses of the study were carried out using Statistical Package for Social Sciences (SPSS) version 24.0 (IBM Corp., Armonk, NY, USA). Since cyclic fatigue resistance data showed normal distribution in all groups, parametric tests were applied. Cyclic fatigue resistance data of each file group (NCF) was analysed by one-way analysis of variance (one-way ANOVA). After ANOVA, post hoc LSD (least significant difference) test was applied to determine the source of the difference between the groups. Data were presented as mean ± standard deviation values. Statistical significance level was determined as *p*  < 0.05. Each analysis was used to determine statistically significant differences between the groups.

## 3. Results

When NFC values were examined among the groups, statistically significant differences were observed as shown in Table 1. PTN (589 ± 63) and PPG (507 ± 51) have significantly higher NFC values compared to ETG (316 ± 45) and FVG (341 ± 71; *p*  < 0.05). Both PTN and PPG and ETG and FVG were statistically similar to each other (*p*  < 0.05).

According to the SEM analyses (Figure 3), areas of initiation of instrument separation for each instrument was shown by arrows. Furthermore, cross section geometry of the groups except ETG was in compliance with the manufacturer's information (Figure 4). ETG represented rectangular and/or round geometric forms.

## 4. Discussion

Fracture due to metallic fatigue occurs in three main stages: crack formation, crack growth, and eventual fracture. This process is usually invisible to the eye as it occurs at the microscopic level [14]. Therefore, investigations on cyclic fatigue behaviours of rotary instrument have great importance for clinical safety and reliability. However, in addition to well-known systems including PTN, several brands of Ni–Ti systems are marketed today. In a review article published in 2018, Gavini et al. [15] reported that more than 160 commercially available systems are present. In the study of Martins et al. [16], they were labelled as “replica-like” instruments. Despite promising results of a number of studies comparing cyclic fatigue resistance of replica-like instruments to that of original brands [17, 18, 19], it is impossible to make a clear judgment on their clinical safety and relevance resulting from abundance. For this purpose, evaluating the most widely used systems in a country or region seems more rational. Thus, the authors of the present study decided to compare the cyclic fatigue resistance of PTN to that of three replica-like instruments; ETG, FVG, and PPG which are the mostly preferred instruments by clinicians in Turkey. The present study is the first study evaluating the cyclic fatigue resistance of contemporary replica-like instruments including PPG, FVG, and ETG.

The results were in line with previous studies [20, 21], which highlighted the effect of cross section design in terms of fatigue resistance. Cross section geometry of both PTN and PPG systems is rectangular. Their offset design allows eccentric rotation and by this way only two corners contact canal walls reducing friction [22]. Combination of M-wire technology and this eccentric motion type may explain both the similarity in their cyclic fatigue resistance and why they are more resistant than ETG and FVG systems which have convex triangular and triangular cross section geometries, respectively. Contact of three points during rotation which is relevant for ETG and FVG systems may have increased friction and reduced fatigue resistance compared to PTN and PPG systems with only two point contact. Thus, our null hypothesis was rejected. Despite the term “Gold” is used in FVG system, the manufacturer defines its production method as AF-R technology. This is also true for ETG which is manufactured from CM-wire but also defined as a gold system. We assume the production information provided by manufacturers for ETG and FVG seems conflicting and questionable because unlike CM and Gold wires, M-wire is a premanufacturing heat treatment [7] and expected to be less resistant compared to Gold and CM-wires resulting from relative high amount of austenite phase in M-wire [23]. Reduced cyclic fatigue resistance of ETG and FVG compared to PTN and PPG may further be related to cross section design/motion style, metallurgic properties resulting from manufacturing methods or both. Furthermore, according to our SEM examinations, ETG instruments represented irregular rectangular or combination of rectangular and round forms diverse from catalogue information which may resulted in increased friction and less cyclic fatigue resistance. On the other hand, comprehensive information on these replica-like systems is either absent or limited. In the study of Ubaed and Bakr [17], AF F-One version of Fanta instruments found to be superior to 2Shape instruments. AF F-One file is also manufactured with AF-R technology as FVG but cross section geometry is S-shaped for AF F-One which provided two point contact to walls and by this way cyclic fatigue resistance may be increased. Also, Plotino et al. [24] revealed that Reciproc instruments with S-shaped cross section providing two point contact have better cyclic fatigue resistance compared to convex triangular-shaped Waveone instruments. Another reason for the difference between PTN–PPG and ETG–FVG systems may be the degree of taper which is regressive for PTG–PPG and constant for ETG–FVG. This situation may also increase friction and reduce cyclic fatigue resistance. The results of the present study and these previous ones are presumably related to the cross section geometry/number of point contacting to canal walls which affects the degree of friction which seems more important than metallurgic properties in terms of cyclic fatigue resistance. In the study of Ates et al. [25], it was reported that rotational speed may inversely affect cyclic fatigue resistance of rotary instruments. However, all systems in the present study were operated at a constant speed and by this way rpm variable could be standardized.

Up to date, various cyclic fatigue test models with different angle of curvature, radius of curvature, and inner diameter were used [26]. Among them test setup used by Larsen et al. [27] with 1.5 mm inner diameter, 60° angle of curvature, and 3 mm radius of curvature were included for the present study. The first reason of selecting this model was the fact stated by Chi et al. [7] which revealed instruments are more prone to fractures in canals with small radius of curvature which is 3 mm for the present study and less than previous studies. This was also supported by Shen et al. [28] who argued that smaller radius of curvatures is one of the most prominent causes of instrument separations. This test model with 1.5 mm simulated canal provides freely rotating of the tested instruments and by this way torsional stresses are ruled out allowing isolated cyclic fatigue evaluation. To ensure standardization, handpiece was attached in a fixed position. A 60° angle of curvature was selected because it is the most frequent degree of canal curvature [29]. Furthermore, preferring dynamic test models could simulate clinical conditions better than static test models. According to previous studies [30, 31, 32], cyclic fatigue resistance of any instruments may either be similar or superior following dynamic testing compared to static test models depending on the type and physical properties of the instruments. Thus, it should be considered that cyclic fatigue values of the instruments included in the present study may vary if tested with a dynamic test model. However, dynamic test designs are incapable of providing reproducibility because of the lack of standardization of the amplitude of axial filing motion [33, 34]. On the other hand, these fatigue test model cannot totally simulate clinical conditions as torsional forces accompany during natural canal instrumentation [18]. In addition, effect of environmental temperature may be either directly or inversely correlated with cyclic fatigue resistance according to the type of instrument [12]. La rosa et al. [35] tested two different file systems at room and body temperature and observed a significant decrease in cyclic fatigue resistance at body temperature. For these reasons, the authors of the present study preferred not to involve temperature change parameter. All test models were set at 35 ± 1°C to simulate human body temperature. Dos Reis-Prado et al. [36] found that the meta-analysis study; NaOCl, especially preheated NaOCl, reduced the cyclic fatigue resistance of some Ni–Ti files. It is possible that the temperature of the solution has a greater effect on fatigue resistance than NaOCl itself. Because the cyclic fatigue of replica-like Ni–Ti files was the main parameter in present study, no heating treatment was applied to NaOCl. Another limitation of the present study is the effect of different pecking motion depths on the dynamic cyclic fatigue resistance of different endodontic instruments which was first study published by La Rosa et al. [37]. They found pecking motions (forward and back movement) improves the cyclic fatigue resistance of the instruments which cannot be simulated with static test models. Improving endodontic instrument durability with specific pecking depths has the potential to improve clinical performance and reduce instrument failures. Furthermore, according to the study of Alajemi and AbuMustafa [38], cyclic fatigue resistance of instruments may be affected by repeated use and sterilization cycles of the instruments. Although they found no impact, another study reported that [39] repeated use of the instruments may have positive effect on cyclic fatigue. Thus, our results need to be verified following repeated use and sterilization cycles.

In this study, cyclic fatigue resistance of different rotary file systems including replica-like instruments were comparatively evaluated to that of PTN with the aim of correlating these features with clinical performance and serving clinicians alternative low price products. This is important to reduce treatment costs for both dentists and patients. Manufacturers often do not provide enough information about their products. Our results represented that PPG seems a safe and effective novel replica-like file system compared to others.

## 5. Conclusion

PTN and PPG can help deliver more reliable and effective treatments by offering higher cyclic fatigue resistance. ETG and FVG groups have lower cyclic fatigue resistance compared to other groups. This shows that these systems may have more limited use under certain conditions. However, it is important to pay attention to canal morphology and needs when selecting files individually for each patient.

## Figures and Tables

**Figure 1:** Metal block for cyclic fatigue test.

**Figure 2:** Handpiece attached to stabilizing arm for static fatigue test.

**Figure 3:** SEM images of the included instruments with ×200 and ×1,000 magnifications: (a) ETG system, (b) FVG system, (c) PPG system, and (d) PTN system.

**Figure 4:** Further surface analysis of instruments belong to ETG group.

**Table 1:** Analysis of the average and standard deviation values of the NCF of the groups.

Groups	Mean	Standard deviation
PTN ^*∗*^	589^a^	63
PPG ^*∗*^	507^a^	51
ETG ^*∗*^	316^b^	45
FVG ^*∗*^	341^b^	71

Different lowercase letters represent significant differences between groups.  ^*∗*^PTN, ProTaper Next;  ^*∗*^PPG, Perfect MTF Plus Gold;  ^*∗*^ETG, EndoArt TouchGold;  ^*∗*^FVG, Fanta V-Taper Gold.

## Data Availability

The findings of this study are supported by data that are available upon request from the corresponding author.
